# Association between Negative Life Events on Mental Health and College Student Adjustment: A Mediated Moderating Effect

**DOI:** 10.1155/2021/4457222

**Published:** 2021-12-20

**Authors:** Liu Cao

**Affiliations:** School of Physical Education, Xuzhou University of Technology, Xuzhou 221018, Jiangsu, China

## Abstract

*Objective*: To explore the association between negative life events and college student adjustment and to explore the mediating and moderating effects of social support and grade level in the relationship between the two. *Methods*. The research was conducted with 1717 college students using the Adolescent Self-Rating Life Events Checklist (ASLEC), China College Student Adjustment Scale (CCSAS), and the Social Support Rating Scale (SSRS). *Results*. (1) Negative life events were significantly negative in correlation with adjustment and social support (*r* = −0.373, −0.174, *Ps* < 0.001), while social support was significantly positive in correlation with adjustment (*r* = 0.359, *P* < 0.001). (2) The main effects of negative life events, social support, and grade on adjustment were significant (effect = −0.190, *P* < 0.001, 95% CI [−0.288∼−0.092]; effect = 0.307, *P* < 0.001, 95% CI [0.265∼0.348]; effect = 0.163, *P* < 0.001, 95% CI [0.126∼0.200]). (3) In the relationship between negative life events and adjustment, social support played a mediating role (effect = −0.054, 95% CI [−0.071∼−0.037]) and grade level played a moderating role (effect = −0.049, *P*=0.009, 95% CI [−0.085∼−0.012]). *Conclusion*. Negative life events, social support, and grade level affected college student adjustment, and social support networks for college students should be actively constructed and targeted education should be conducted according to different grade levels, which can promote college student adjustment.

## 1. Introduction

Adjustment was primarily a response to psychosocial stressors or multiple stressors and is an important dimension of mental health. From a global mental health perspective, typical triggering stressors for adjustment problems are economic hardship, forced migration, and loss of resources due to adjustment to a new environment or culture [1]. But adjustment problems, particularly adjustment disorders, have long been neglected in mental health research. At present, technological developments have led to a much faster pace of social development, adjustment is becoming an increasing concern, and adjustment disorders have become a common diagnosis in clinical practice worldwide [2]. Adjustment among university students has also gradually become an emerging issue [3] and has become one of the important criteria for measuring the mental health of university students. Adjustment has unique characteristics, not only in terms of adjustment to school but also in terms of adjustment to career choice and social adjustment. The impact of these factors on college students is a large proposition that requires systematic and comprehensive research, and the factors that influence adjustment have become an important area of concern for researchers. Among the influences on adjustment, negative life events or stressful events are globally recognized and proven influencers [4]. In terms of the national and international literature searched for in the study, there is less empirical evidence on adjustment among university students, which is one of the main reasons and innovations for the conduct of this study.

Adjustment is strongly associated with life events. Apart et al. stated that individuals faced with significant negative life events (e.g., death of a loved one, loss of employment, and environmental change) invariably experience adjustment problems, leading to a range of mental health problems [5]. The experience of stressful life events can lead to problems in psychological adjustment (e.g., depression and life satisfaction) [6]. More seriously, if faced with higher levels of stress or after experiencing a traumatic life event, this may be accompanied by stress disorders or adjustment disorders and serious mental health problems [7]. Studies have found that stressful events are significant predictors of adjustment disorders [8]. The DSM-5 states that adjustment disorders have significant event triggers and are accompanied by significant emotional and behavioural symptoms [9]. It is evident that adjustment due to negative life events or negative life experiences is a relatively common mental health problem [10, 11].

In addition, adjustment problems occur in all cultures and can occur at any age, with a high prevalence in the general population [12], but not enough attention has been paid to adjustment disorders [13]. Mcgue and Bouchard noted that for most psychological and physiological variables, age and gender have a strong influence [14]. A meta-analysis by Roorda et al. found that age (expressed by grade level) was a moderating variable for attachment and school adjustment [15]. Lei et al. also found that age moderated the relationship between teacher-student relationships and students' externalising behaviours, with the upper primary school student group being stronger than the other student groups [16]. Some studies further suggest that age plays a moderating role in parental rejection acceptance and adjustment, with younger children perceiving more rejection from their parents and showing more negative emotions compared to older children [17]. Analysis of the literature suggests that mechanisms for the role of age in adjustment are stable, but are more theoretical and have relatively few empirical findings. Even fewer have explored the moderating role of age with respect to the relationship between life events and adjustment. Relatively few studies have been conducted on university students in the 19–23 age group, who are enrolled in four years, freshman through senior year. The mechanism of the role between grades is one of the innovations of this study. Accordingly, this study proposes hypothesis 1: grade level plays a moderating role in the relationship between negative life events and adjustment.

Among the influencing factors of mental health, social support has been considered as the more stable influencing variable [18, 19]. The buffering model of social support states that adequate support can buffer the effects of stressful events on adverse outcomes and promote emotional and behavioural adjustment and that social support is an important influential variable between stressful events and adjustment [20]. Similarly, the phenomenological variant of ecological systems theory (PVEST) as a theoretical framework explains the role of social support. The PVEST focuses on the ecosystem in which the individual grows, emphasising the development and adaptation of the individual in terms of macrosystems, mesosystems, and microsystems. This theory emphasises the coping and adaptive processes of individuals in resource acquisition, coping, and adaptation directly influence individual-related behaviour and health. PVEST considers social support as an important protective factor that can influence the relationship between stressful events and outcomes [21]. In terms of the overall function of social support, researchers have noted that higher levels of social support influence the relationship between stressful life events and behavioural adjustment [22], while others have identified a mediating role of social support between negative life events and depression and suicidal ideation [23, 24]. Some have explored the role of social support in terms of specific types of social support, with Anne and Carleton noting that the more negative life events an individual experiences and the lower the perceived parental support, the more severe the adjustment problems, which can lead to an increased risk of depression and internalising and externalising behavioural problems [25]. Others have found that sibling support reduces the association between negative life events and maladjustment [26, 27]. In addition, researchers have noted that perceived support is more important than received support in predicting adjustment to stressful life events [28]. The above studies affirm the mediating role of social support between negative life events and adjustment. A literature search revealed few relevant studies and even fewer studies on Chinese university students. Based on this, this study proposed hypothesis 2: social support is a mediating variable in the relationship between negative life events and college students' adjustment, taking Chinese college students as the target population.

According to hypothesis 1 and hypothesis 2, the study constructs a mediated moderating model in the relationship between negative life events and college students' adjustment, with the moderating variable being grade level and the mediating variable being social support. The model diagram is shown in Figure 1.

## 2. Methods

### 2.1. Participants

A completely random sample of university students from six undergraduate colleges in Jiangsu Province was used. The study was approved by the ethics committee of the college, and the subjects were informed of the purpose of the study and signed an informed consent form before the survey. A total of 1852 questionnaires were distributed and 1806 were returned, with a return rate of 97.5%; the final number of valid subjects was 1717, with an effective rate of 95.1%. Among the valid subjects, 875 (51%) were males and 842 (49%) were females; 495 (28.8%) were freshmen, 454 (26.4%) sophomores, 410 (23.9%) juniors, and 358 (20.9%) seniors.

### 2.2. Measures

#### 2.2.1. Adolescent Self-Rating Life Events Checklist (ASLEC)

The Adolescent Self-Rating Life Events Checklist (ASLEC) was developed by Liu and Liu and was used to measure negative life events among university students [29]. The questionnaire mainly consisted of 27 negative life events that may bring about psychophysiological reactions in adolescents, including six factors such as interpersonal relationships, academic stress, being punished, loss of family, friends and possessions, health adjustment, and others. Each event should be answered in such a way that the occurrence of the event within a limited period of time is determined first. If it did not occur, a score of 0 is assigned, and if it did occur, it is rated on a 5-point scale (1 for no, 2 for mild, 3 for moderate, 4 for severe, and 5 for very severe) according to the psychological feelings at the time of the event, with higher scores indicating a greater number of negative life events experienced and a greater impact. The Cronbach's alpha coefficient for the questionnaire was 0.85 and the corrected half reliability coefficient was 0.88. The Cronbach's alpha coefficient for the total questionnaire in this study was 0.88. The scale was widely used in related studies in China and the construct validity has been further validated.

#### 2.2.2. China College Student Adjustment Scale (CCSAS)

The China College Student Adjustment Scale (CCSAS) was developed by Fang Xiaoyi and was used to measure the adjustment of college students [30]. The questionnaire mainly consisted of 60 questions, including 7 factors such as interpersonal adjustment, study adjustment, campus adjustment, career choice adjustment, emotional adjustment, self-adjustment, and satisfaction. A Likert 5-point scale was used, ranging from 1 = disagree to 5 = agree, with the higher the score, the better the adjustment. The Cronbach's alpha coefficient for the questionnaire was 0.93 and the 7-factor Cronbach's alpha coefficient ranged from 0.65 to 0.82. The Cronbach's alpha coefficient for the total questionnaire in this study was 0.96. The results of the exploratory factor analysis and validation factor analysis indicate that the scale has good construct validity.

#### 2.2.3. Social Support Rating Scale (SSRS)

The Social Support Rating Scale (SSRS) developed by Xiao was used to measure the social support of university students [31]. The questionnaire consisted of 10 questions, including 3 factors: subjective support, objective support, and the degree of use of support. The higher the score on the questionnaire, the better the social support. The scale retest reliability was 0.92. The scale is one of the most widely used tools in China, and its validity has been verified.

### 2.3. Procedures

The tests were administered by graduate students and counsellors in psychology, all of whom were systematically trained in measurement before testing and carried out after passing the training. Participants did not know the purpose of the test before testing. The tests were administered in class groups and were controlled to last about 30 minutes. All questionnaires were distributed on the spot and collected on the spot. A fee is paid for the completion of the answer. The recovered questionnaires were checked and then a database was created and the data were analysed and processed using SPSS 27.0, Excel, and the macroprogram Process developed by Hayes. Mean scores and standard deviations for negative life events, adjustment, and social support were analysed using descriptive statistics. Pearson product-difference correlations were used to analyse the correlation between negative life events, adjustment, social support, and grade level. Mediating and moderating effects were analysed using Process, a macroprogram developed by Hayes, using the bootstrap method, with a sample of 5000 and a significance test of 95%.

## 3. Results

### 3.1. Descriptive Statistics and Correlation Analysis of the Variables

Correlation analysis of the study variables found (Table 1) that negative life events were significantly negatively correlated with adjustment and social support (*r* = −0.373, −0.174, Ps < 0.001) and social support was significantly positively correlated with adjustment (*r* = 0.359, *P* < 0.001). The correlation between grade and negative life events and adjustment was low, and negative life events were more strongly correlated with adjustment, with grade acting as a moderating variable according to the MacArthur method criteria [32], in line with the study hypothesis. The MacArthur method criteria is that intermediate variables, predictor variables, and outcome variables are significantly correlated and predictor variables are not correlated or are less correlated with intermediate variables, which can be judged as moderating variables.

### 3.2. The Association between Negative Life Events and College Student Adjustment: A Mediated Moderating Effect

In conjunction with the prior hypotheses, the conditions for conducting a moderated model test were met according to the structural equation modeling approach [33] and the results of the correlation analysis, so the mediating role of social support and the moderating role of grade level were examined in the relationship between negative life events and adjustment. The analyses were conducted using Process, a macroprogram developed by Hayes. Negative life events, adjustment, and social support were first standardised and then tested for mediated moderating effects.

The mediating effect of social support in the relationship between negative life events and adjustment was first analysed (Table 2). The main effects of negative life events and social support on adjustment were all significant (effect = −0.190, *P* < 0.001, 95% CI [−0.288 to −0.092]; effect = 0.307, *P* < 0.001, 95% CI [0.265 to 0.348]), as was the main effect of negative life events on social support (effect = −0.174, *P* < 0.001, 95% CI [−0.220 to −0.127]). A mediating effect of social support in the relationship between negative life events and adjustment is valid (effect = −0.054, 95% CI [−0.071 to −0.037]). The mediating effect of social support in the relationship between negative life events and adaptation is established.

More importantly, the main effect of grade on adjustment was significant (effect = 0.163, *P* < 0.001, 95% CI [0.126 to 0.200]) and the effect of grade interacting with negative life events on adjustment was also significant (effect = −0.049, *P*=0.009, 95% CI [−0.085 to −0.012]), with grade playing a significant role in the relationship between negative life events and adjustment. The moderating effect of grade level in the relationship between negative life events and adjustment holds true. To gain a clearer understanding of the moderating effect of grade level, a simple slope test was conducted to examine the effect of negative life events on adjustment across the four grades and a simple effect analysis was plotted. The results of the test (Figure 2) show that for all four grades, negative life events were a significant negative predictor of adjustment, with the fourth grade adjustment score being the highest and the first grade adjustment score being the lowest in the low negative life event group, while in the high negative life event group, the first grade adjustment score was the highest and the fourth grade adjustment score was the lowest. That is, the lower the number of negative life events experienced and the higher the grade level, the better the adjustment, while the higher the number of negative life events experienced and the higher the grade level, the worse the adjustment.

## 4. Discussion

This study found that negative life events were significantly and negatively associated with adjustment, suggesting that the more negative life events experienced by college students, the more likely they are to have problems with adjustment. There is growing evidence that adjustment may be related to stressful life events and may occur after exposure to traumatic events [4]. A study by Mahat-Shamir et al. found that exposure to stressful or traumatic events within the past month was significantly associated with symptoms of adjustment disorder (ICD-11) and that previous traumatic events may be a risk factor for adjustment disorder [34]. In terms of specific symptoms, individuals who experience negative life events exhibit more internalising problems (depression and anxiety) [35]. Studies with adolescents have found a greater association between life events and adolescent adjustment [36, 37], and these validate the present study. Negative life events can lead to changes in individual, family, and school life, which in turn can interfere with and disrupt adolescents' adaptive functioning. In addition, there is a relationship between adolescents' adjustment and the number of negative life events, with higher numbers also predisposing adjustment to problems [38].

Consistent with our hypothesis, the present study found that social support mediated the relationship between negative life events and adjustment. The results validate the stress buffer effect model of social support. The stress buffering effect model states that higher social support as well as problem-solving skills buffer the adverse effects of stressful events on emotional/behavioural problems. As previously mentioned, Waite et al. found that sibling support reduced the association between negative life events and maladjustment [27], which supports the buffering effect model, whereas individuals experiencing negative life events are more or less likely to have adjustment problems and social support alleviates the tension and frustration that individuals experience as a result of the event and increases their confidence to deal with the problem as well as to adopt effective coping to avoid emotional/behavioural problems. It is evident that the stronger the social support network one has, the better one is able to cope with challenges from a variety of sources. The role of social support is crucial in the Chinese cultural context, where university students who experience negative or stressful life events receive more support from school and family, as well as from friends or peers. Each year, during the new student intake and college graduation season, education departments and schools conduct targeted school adjustment and social adjustment education to guide students in their new environment.

The study further explored the moderating effect of grade level in the relationship between negative life events and adjustment and found that negative life events had a significant predictive effect on adjustment in all four grade levels. The high grouping of negative life events resulted in the best adjustment in grade 1 and the worst adjustment in grade 4; the low grouping of negative life events resulted in the best adjustment in grade 4 and the worst adjustment score in grade 1. In the normal life state (low negative or stressful life events), the older the age, the better the adjustment. Adjustment in this study was more of an adjustment to university life. Senior university students had already had more experiences and experiences of university life and were faced with minor setbacks and problems that they were able to handle better, which facilitated their adjustment. Similarly, university students are faced with new decisions or pressures, such as the pressure to choose a career and the pressure to graduate. In contrast, senior students have a much higher stress index and experience of stress than junior students and therefore may briefly show many discomforts, while junior students experience these temporarily less deeply and have fewer adjustment problems.

Therefore, this study proposes a model of mediated moderating effects based on a buffering effect model of social moderating and a theory of adjustment barriers, addresses the relationship between negative life events and adjustment, and identifies the role of grade level and social support in the relationship between the two. It was found that negative life events produced greater predictors of adjustment among Chinese university students and that grade level showed some differences in the number of negative life events, with social support being an important mediating factor. The results enrich the study of the relationship between negative life events and adjustment using a Chinese sample and are important for guidance and application in the development of adjustment education for university students across grade levels based on a social support perspective. The data source for this study is a cross-sectional study, and if further exploration of the relationships is needed, longitudinal research is a future endeavour, which is a limitation of this study.

## Figures and Tables

**Figure 1:** The association between negative life events and college student adjustment: a mediated moderating effect.

**Figure 2:** Simple slope plot of the association between negative life events and college student adjustment under grade moderation.

**Table 1:** Descriptive statistics and correlation matrix of the variables (*n* = 1717).

	M	SD	NLE	CSA	SS	GR
1. NLE	1.29	0.57	1			
2. CSA	3.57	0.37	−0.373^*∗∗∗*^	1		
3. SS	38.69	6.34	−0.174^*∗∗∗*^	0.359^*∗∗∗*^	1	
4. GR	——	——	−0.061^*∗*^	0.194^*∗∗∗*^	−0.014	1

*Note.* ^*∗*^ *p* < 0.05, ^*∗∗∗*^*p* < 0.001. NLE = negative life events; SS = social support; GR = gender; CSA = college student adjustment.

**Table 2:** The association between negative life events and college student adjustment: a mediated moderating effect.

SS		CSA				
	Effect	*t*	Effect	*t*	LLCI	ULCI
NLE	−0.174	−7.307^*∗∗∗*^	−0.190	−3.789^*∗∗∗*^	−0.288	−0.092
SS			0.307	14.547^*∗∗∗*^	0.265	0.348
GR			0.163	8.675^*∗∗∗*^	0.126	0.200
NLE ^*∗*^ GR			−0.049	−2.624^*∗∗*^	−0.085	−0.012
*R* ^*2*^ = 0.030,*F*(1,1715) = 53.398, *P* < 0.001			*R*2 = 0.264, *F*(4,1712) = 153.300, *P* < 0.001 R2-chng = 0.003, *F*(1,1712) = 6.887, *P*=0.009			

*Note.* ^*∗*^ *p* < 0.01, ^*∗∗∗*^*p* < 0.001. NLE = negative life events; SS = social support; GR = gender; CSA = college student adjustment.

## Data Availability

The data used to support the findings of this study are available from the corresponding author upon request.
